# VEGF Family Gene Expression as Prognostic Biomarkers for Alzheimer's Disease and Primary Liver Cancer

**DOI:** 10.1155/2021/3422393

**Published:** 2021-11-20

**Authors:** Kai Xu, Chuan-ling Wu, Zhi-xin Wang, Hai-jiu Wang, Feng-jiao Yin, Wen-deng Li, Chu-chu Liu, Hai-ning Fan

**Affiliations:** ^1^Department of Hepatopancreatobiliary Surgery, Affiliated Hospital of Qinghai University, China; ^2^Jianhu College, Zhejiang Industry Polytechnic College, China; ^3^Qinghai Province Key Laboratory of Hydatid Disease Research, China

## Abstract

**Background:**

To analyze the expression of vascular endothelial growth factor (VEGF) in hepatocellular carcinoma (HCC) and cognitive impairment, explore the relationship between the expression of VEGF family genes and prognosis of patients with HCC, and evaluate the predictive ability of VEGF in cognitive impairment using computerized methods.

**Methods:**

VEGF expression in liver cancer tissues and normal tissues was analyzed using bioinformatics methods. The Kaplan-Meier survival analysis method was also used to analyze the relationship between VEGF expression and the prognosis of patients with HCC. Furthermore, immune infiltration assessment and gene set enrichment analysis were performed. Meanwhile, the differential expression of VEGF family genes between patients with Alzheimer's disease (AD) and healthy controls was also checked.

**Results:**

Based on The Cancer Genome Atlas (TCGA) database, the VEGF family genes (*VEFGA*, *VEGFB*, *VEGFC*, and *VEGFD*) were highly expressed in cancer tissues and were significantly associated with poor prognosis in HCC. In HCC, the VEGF family genes showed significant heterogeneity in their functional and immune infiltration characteristics. Finally, VEGF family genes were identified as prognostic biomarkers in AD and risk prediction markers in HCC.

**Conclusions:**

VEGF is highly expressed in patients with HCC and lowly expressed in patients with AD. VEGF has opposite opposing roles in the treatment of tumors and cognitive impairment.

## 1. Introduction

Liver cancer is the most common fatal malignancy and is the fourth leading cause of cancer-related deaths worldwide [1, 2]. Globally, liver cancer accounted for 1 million cases and 829,000 deaths in 2016 [3]. Liver cancer is more common in males, with 1 in 38 men developing liver cancer compared to 1 in 111 females [3]. More than 90% of all liver cancer cases are those of hepatocellular carcinoma (HCC), for which chemotherapy and immunotherapy are currently the best treatment options [4]. Older age and associated comorbidities and cognitive impairment are detrimental factors affecting therapeutic interventions in cancer [5]. Older patients tend to be more reluctant to undergo surgery because of various reasons, such as frailty. The prevalence of MCI is 10 to 20% in adults aged 65 years and older, with the risk of cognitive impairment increasing with age [6].

Previous studies have shown that HCC is a vascular endothelial growth factor- (VEGF-) driven tumor [7]. The blood supplies nutrients to the tumor cells for growth and invasion and also helps in getting rid of metabolic wastes. A study showed that plasma VEGFA levels were decreased in patients with mild cognitive impairment [8]. Other studies have shown that VEGFs ameliorate cognitive impairment [9]. Therefore, VEGF plays a complex role in both tumor development and cognitive impairment progression. However, the role of VEGF in the context of HCC and cognitive impairment remains unclear.

The availability of genome sequencing data for many diseases has facilitated the application of bioinformatics methods to the study of molecular associations between different diseases. In this study, we applied a bioinformatics approach to investigate the possible role of VEGF in patients with HCC and cognitive impairment. This study provides new insights into the treatment of patients with HCC and cognitive impairment.

## 2. Materials and Methods

### 2.1. Data Acquisition and Differential Gene Expression Analysis

Transcriptomic data and clinical data of patients with HCC were downloaded from The Cancer Genome Atlas (TCGA) database (https://portal.gdc.cancer.gov). The human cognitive impairment-related dataset GSE140831 was obtained from the Gene Expression Omnibus (GEO) database. The GSE140831 dataset included blood transcriptomic data of 530 normal controls and 204 patients with AD. The limma package in R language was used to perform differential expression analysis (high versus low expression) of VEGF family genes in tumor and normal tissues. The limma package was also used to perform differential expression analysis of genes in the blood of healthy controls and patients with cognitive impairment. All data were saved in text form.

### 2.2. Gene Set Enrichment Analysis (GSEA)

To identify VEGF family gene-related signaling pathways, GSEA was performed using GSEA v4.0.3, based on the HCC prognosis-related gene set in the Molecular Signatures Database (MSigDB). The HCC prognosis-related gene set in MSigDB was used as the reference gene set, and other parameters were set based on default values.

### 2.3. Immune Infiltration Assessment

The algorithm for the assessment of immune cell infiltration was established using the GSVA package of R software (version 3.6.3). RNA sequencing (RNA-Seq) data were obtained in the HTSeq-FPKM format, and clinical data were obtained from the liver hepatocellular carcinoma (LIHC) project. Paracancerous tissues were excluded from the analysis.

### 2.4. Statistical Analysis

Statistical analysis was performed using GraphPad Prism 6.0 software and R software (version 3.6.3). The mRNA levels of VEGF family genes in HCC and normal tissues were compared by *t*-test. The Kaplan-Meier method was applied for survival analysis, and the log-rank test was used to assess differences in survival curves. The survival receiver operating characteristic (ROC) package in R software was used to plot ROC curves, and the area under the curve (AUC) was also calculated to assess the predictive accuracy of the model. The model was considered to have good predictive power when AUC > 0.7. Finally, univariate Cox regression analysis of VEGF family genes and clinical characteristics was performed to assess the prognostic value of each VEGF family gene.

## 3. Results

### 3.1. Prognostic Features of VEGF Family Genes in Hepatocellular Carcinoma

Based on the TCGA database, vascular endothelial growth factor (VEGF) family genes (*VEFGA*, *VEGFB*, *VEGFC*, and *VEGFD*) were highly expressed in cancer tissues (Figure 1(a)). Survival analysis suggested that the high expression of VEGF family genes was significantly associated with poor prognosis in all cases of HCC (Figure 1(b)). Characterization of VEGF in HCC tissues showed that the T stage of the tumor was significantly correlated with the expression of *VEGFA* and *VEGFB* but not with that of *VEGFC* and *VEGFD* (Table 1). In addition, age was also found to be significantly correlated with the expression of *VEGFB* (Table 1). A similar finding was found in the univariate Cox analysis of the expression of VEGF family genes in HCC (Table 2). The expression of *VEGFA* was associated with the T stage, pathologic stage, and sex; the expression of *VEGFB* was associated with the T stage, pathologic stage, sex, age, body mass index (BMI), alpha-fetoprotein (AFP) level, and albumin level; the expression of *VEGFC* was only associated with the Child-Pugh grade; and the expression of *VEGFD* was associated with the age and pathologic stage. These results suggest that the expression of all VEGF family genes is associated with liver cancer prognosis; however, each gene may play different functions. Therefore, VEGF family genes may serve as prognostic biomarkers for liver cancer.

### 3.2. Functional Characterization and Immune Infiltration of VEGF Family Genes in HCC

GSEA suggested that the *VEGFA* gene was significantly enriched in the Focal Adhesion PI3K AKTMTOR Signaling Pathway gene set (*P* adjust = 0.029; false discovery rate [FDR] = 0.023) and the Reactome Extracellular Matrix Organization gene set (*P* adjust = 0.029; FDR = 0.023) (Figure 2(a)). The *VEGFA* gene was not significantly enriched in the Binding gene set (*P* adjust = 0.062; FDR = 0.052) and Reactome M Phase (*P* adjust = 0.062; FDR = 0.052) (Figure 2(b)). The *VEGFC* gene was significantly enriched in the Reactome Neutrophil Degranulation gene set (*P* adjust = 0.013; FDR = 0.009) and the Reactome GPCR Ligand Binding gene set (*P* adjust = 0.013; FDR = 0.009) (Figure 2(c)). The *VEGFD* gene was significantly enriched in the Reactome Biological Oxidations gene set (*P* adjust = 0.124; FDR = 0.114) but not in the Reactome SLC Mediated Transmembrane Transport gene set (*P* adjust = 0.124; FDR = 0.114) (Figure 2(d)). This suggests that VEGF family genes are involved in different pathways and perform different functions. The immune infiltration analysis regarding VEGF family gene expression revealed that VEGF family genes phenotypically exhibit immune infiltration-related heterogeneity (Figures 3(a)–3(d)). In conclusion, the functional characteristics of VEGF family genes exhibit significant heterogeneity with respect to immune infiltration characteristics.

### 3.3. VEGF Family Genes Collectively Constitute a Prognostic Biomarker for Liver Cancer

Pearson's correlation analysis of the expression of VEGF family genes in liver cancer tissues suggested a significant positive correlation between the expression of *VEGFA*, *VEGFB*, and *VEGFC* with different patient characteristics and tumor properties, such as the pathologic stage, age, sex, BMI, and AFP and albumin levels (Figures 4(a) and 4(b)). Unexpectedly, no significant correlation was found between the expression of VEGF family genes and vascular infiltration (Figure 4(c)). The AUC curves of VEGF family genes and liver cancer prognosis suggested that all VEGF family genes could be used as biomarkers to evaluate the prognosis of patients with liver cancer (Figure 4(d)).

### 3.4. VEGF Family Genes Collectively Constitute a Biomarker for AD Risk

In this study, VEGF family genes were significantly downregulated in the blood of patients with AD (Figure 5(a)). Results of AD-related functional characteristics and GSEA are shown in Figure 5(b). The AUC curve showed that the expression of VEGF family genes (*VEGFA*, *VEGFB*, and *VEGFC*) was associated with AD risk (Figure 5(c)). Correlation analysis of the expression of VEGF family genes in the blood of patients with AD suggested a significant positive correlation between the expression of *VEGFA*, *VEGFB*, and *VEGFC* with AD risk (Figure 5(d)). Additionally, the VEGF family genes, including *VEGFA*, *VEGFB*, and *VEGFC*, together displayed good predictive power (AUC = 0.756) for AD risk (Figure 5(e)). The expression profiles of VEGF family genes, including *VEGFA*, *VEGFB*, and *VEGFC*, in healthy controls and patients with AD are shown in Table 3.

## 4. Discussion

The development and invasion of HCC are closely related to the revascularization of the primary tumor. Neovascularization provides oxygen and nutrients required for tumor cell proliferation while removing metabolic waste products. The VEGF family plays a vital role in proangiogenesis and drives various oncogenic processes, such as cell proliferation, migration, differentiation, and cytoskeletal reorganization. Overexpression of VEGF is associated with accelerated tumor progression and poor prognosis in various cancers, including breast, lung, gastric, and colorectal cancers [10]. Similarly, VEGF plays a complex role in the development of cognitive impairment. One study found decreased levels of plasma VEGFA in patients with mild cognitive impairment [8]. Interestingly, another study showed an increased expression of VEGF in patients with mild cognitive impairment [11]. Taken together, these findings demonstrate the complex role of VEGF in the development of HCC and neurodegenerative diseases. In this study, we showed the role of four VEGF family members, namely, VEGFA, VEGFB, VEGFC, and VEGFD, in HCC and cognitive impairment by analyzing their gene expression in patients with HCC and patients with AD. Differential gene expression analysis revealed that the expression of VEGF family genes was elevated in patients with HCC and decreased in patients with AD. Survival analysis further showed that higher expression of VEGF was associated with a worse prognosis.

Human HCC is a VEGF-driven tumor that relies on the blood supply for nutrients and to eliminate metabolic wastes [7]. In line with this, our results showed the upregulation of *VEGFA*, *VEGFB*, *VEGFC*, and *VEGFD* genes in patients with HCC compared to healthy controls. Hypoxia-inducible factor-1*α* (HIF-1*α*) and survivin can promote hepatic tumor angiogenesis by upregulating VEGF protein expression, thereby accelerating hepatocarcinogenesis and progression [12, 13]. Another study found that microRNA-26b could inhibit liver tumor growth by suppressing the NF-*κ*B/MMP-9/VEGF pathways [14]. In addition, melatonin can interfere with the transcriptional activation of VEGF via HIF-1*α* and STAT3, thus exerting an antiangiogenic effect on liver tumors [15] and ultimately inhibiting tumor growth. Our study showed that the upregulation of VEGF family genes was associated with shorter overall survival and worse prognosis in patients with HCC.

VEGF, which promotes lymphovascular repair and regeneration, increased blood-brain barrier (BBB) permeability, and mild neuroprotection is gaining increasing attention in the treatment of cognitive impairment [16]. A previous study has found decreased levels of plasma VEGFA in patients with mild cognitive impairment [8]. The same trend was also observed in our analysis. Moreover, we found that VEGFA, VEGFB, and VEGFC were all downregulated in patients with AD and that each of them could independently predict the risk of developing AD. However, one study showed the elevation of plasma VEGF in patients with mild cognitive impairment [11]. Another study analyzed transcriptomic data from the prefrontal cortex of patients with cognitive impairment and found that high VEGFB expression was associated with an unsatisfactory cognitive performance [17]. Alvarez et al. suggested that VEGF expression may be endogenously increased due to several pathological factors, which may have a protective effect on cognition in patients with AD [9]. In obese mice, a compensatory increase in VEGF expression restored glucose metabolism, which in turn preserved cognition and minimized the deleterious effect of neurodegenerative lesions [18]. Increased VEGF/VEGF-A expression restored cerebral vasculature and promoted the regeneration of neuronal structures, synapses, and nerves in mice, thereby improving cognitive dysfunction [19]. Additionally, VEGFC plays an essential role in the development of meningeal lymphatic vessels (MLV) [20]. In aged mice, VEGFC enhanced the meningeal lymphatic drainage of macromolecular metabolic wastes in the cerebrospinal fluid, resulting in improved cognition [21]. A recent clinical trial showed that the combination of anti-VEGF and anti-PD-L1 therapies prolongs progression-free survival in patients with unresectable HCC [22]. This confirms that antiangiogenesis therapy, especially anti-VEGF therapy, can be helpful in the treatment of HCC. However, anti-VEGF therapy may cause cognitive impairment by damaging neurons as well as inhibiting neovascularization [23–25]. Therefore, future studies should focus on strategies to efficiently apply antiangiogenic therapy without inducing cognitive impairment in patients.

Currently, antiangiogenesis therapy has emerged as an effective alternative to chemotherapy in the treatment of cancer. Although antiangiogenesis therapy provides some benefit to patients with HCC, the effects remain unsatisfactory. Furthermore, given the protective role of VEGF in cognitive impairment, the antiangiogenic effect may cause impairment of cognitive function and further exacerbation of neurodegenerative lesions in patients. In our study, we implemented a bioinformatics approach to provide a comprehensive account of the role of VEGF in HCC and cognitive impairment. First, we determined that VEGF expression was upregulated in HCC tissues compared to normal tissues. Next, we confirmed that elevated VEGF levels led to worse overall survival in patients with HCC. Finally, we found that VEGF expression was associated with AD; lower expression of VEGF was associated with a higher occurrence of AD. These results suggest that VEGF acts as a double-edged sword, protecting against cognitive impairment while promoting tumor development and decreasing the overall survival of patients.

The present study also has some limitations. First, this study failed to directly analyze the role of VEGF in the relationship between HCC and AD. Second, further experimental verification was lacking. Third, there is a lack of relevant clinical follow-up cases for the validation of VEGF as a prognostic and predictive biomarker. In a word, more experimental studies need to be added in the future.

Neurovascular-related diseases and genes have been extensively studied over the years [26, 27]. Coupled with an ever-increasing amount of bioinformatics tools, Bioinformatics is playing an increasingly important role [28, 29]. In this study, we illustrated the double-edged effect of VEGF in HCC and AD; VEGF expression leads to poor prognosis in HCC while it plays a protective role in cognition. Therefore, it is critical to developing proper strategies for the application of antiangiogenesis therapies in patients with cancer, especially elderly patients with HCC who are more prone to cognitive impairment. Future studies should focus on the development and application of antitumor angiogenic therapy, which does not result in cognitive damage to patients.

## 5. Conclusion

Using bioinformatics methods, we illustrated that VEGF has opposing roles in the treatment of tumors and cognitive impairment. Future studies could focus on the efficient use of antitumor angiogenesis therapy to reduce or avoid cognitive impairment in patients. In this way, the quality of life in patients with liver cancer can be significantly improved with a better prognosis.

## Figures and Tables

**Figure 1:** Prognostic features of vascular endothelial growth factor (VEGF) family genes in hepatocellular carcinoma. (a) Differential expression of VEGF family genes (*VEFGA*, *VEGFB*, *VEGFC*, and *VEGFD*) in cancer and normal tissues. (b) Expression and survival analysis curves of VEGF family genes (*VEFGA*, *VEGFB*, *VEGFC*, and *VEGFD*).

**Figure 2:** Functional characterization and gene set enrichment analysis (GSEA) of vascular endothelial growth factor (VEGF) family genes, including *VEGFA* (a), *VEGFB* (b), *VEGFC* (c), and *VEGFD* (d).

**Figure 3:** Functional characteristics and immune infiltration characteristics of VEGF family genes. Immune infiltration analysis suggested that VEGF family genes, including *VEGFA* (a), *VEGFB* (b), *VEGFC* (c), and *VEGFD* (d), phenotypically exhibit immune infiltration-related heterogeneity. Notes: aDC: activated DC; iDC: immature DC; pDC: plasmacytoid DC; Tcm: T central memory; Tem: T effector memory; Tfh: T follicular helper; Tgd: T gamma delta.

**Figure 4:** VEGF family genes collectively constitute a prognostic biomarker for liver cancer. (a, b) Correlation analysis of VEGF family gene expression in hepatocellular carcinoma tissues. (c) Correlation of VEGF family genes with tumor vascular infiltration. (d) AUC curves of VEGF family genes were correlated with liver cancer prognosis.

**Figure 5:** VEGF family genes collectively constitute a predictive biomarker for AD. (a) Differential expression of VEGF family genes (*VEFGA*, *VEGFB*, and *VEGFC*) between healthy controls and patients with AD. (b) AD-related functional characterization and GSEA enrichment analysis. (c) AUC curves of VEGF family genes (VEGFA, VEGFB, and VEGFC) were associated with AD risk. (d) Correlation analysis of the expression of VEGF family genes (*VEGFA*, *VEGFB*, and *VEGFC*) in blood with AD risk. (e) ROC curves suggest that the VEGF family genes (*VEGFA*, *VEGFB*, and *VEGFC*) collectively constitute a predictive biomarker for AD.

**(a):** 

Characteristic	VEGFA			VEGFB		
	Low expression	High expression	*P* value	Low expression	High expression	*P* value
Number	187	187		187	187	
T stage, *n* (%)			0.035			0.031
T1	103 (27.8%)	80 (21.6%)		105 (28.3%)	78 (21%)	
T2	47 (12.7%)	48 (12.9%)		40 (10.8%)	55 (14.8%)	
T3	30 (8.1%)	50 (13.5%)		33 (8.9%)	47 (12.7%)	
T4	5 (1.3%)	8 (2.2%)		6 (1.6%)	7 (1.9%)	
N stage, *n* (%)			0.623			0.123
N0	124 (48.1%)	130 (50.4%)		124 (48.1%)	130 (50.4%)	
N1	1 (0.4%)	3 (1.2%)		0 (0%)	4 (1.6%)	
M stage, *n* (%)			1.000			0.126
M0	134 (49.3%)	134 (49.3%)		126 (46.3%)	142 (52.2%)	
M1	2 (0.7%)	2 (0.7%)		0 (0%)	4 (1.5%)	
Age, median (IQR)	59.5 (51, 68)	62 (54, 69)	0.143	63 (54.5, 69)	60 (50, 68)	0.029

**(b):** 

Characteristic	VEGFC			VEGFD		
	Low expression	High expression	*P* value	Low expression	High expression	*P* value
Number	187	187		187	187	
T stage, *n* (%)			0.635			0.190
T1	89 (24%)	94 (25.3%)		101 (27.2%)	82 (22.1%)	
T2	52 (14%)	43 (11.6%)		45 (12.1%)	50 (13.5%)	
T3	41 (11.1%)	39 (10.5%)		33 (8.9%)	47 (12.7%)	
T4	5 (1.3%)	8 (2.2%)		7 (1.9%)	6 (1.6%)	
N stage, *n* (%)			0.622			1.000
N0	125 (48.4%)	129 (50%)		129 (50%)	125 (48.4%)	
N1	1 (0.4%)	3 (1.2%)		2 (0.8%)	2 (0.8%)	
M stage, *n* (%)			0.361			1.000
M0	138 (50.7%)	130 (47.8%)		139 (51.1%)	129 (47.4%)	
M1	1 (0.4%)	3 (1.1%)		2 (0.7%)	2 (0.7%)	
Age, median (IQR)	62 (52, 69)	60 (51, 68)	0.394	59 (51, 68)	64 (53, 69)	0.053

**(a):** 

Characteristics	VEGFA		VEGFB	
	Odds ratio (OR)	*P* value	Odds ratio (OR)	*P* value
T stage (T2 & T3 & T4 vs. T1)	1.664 (1.106-2.514)	0.015	1.857 (1.232-2.811)	0.003
N stage (N1 vs. N0)	2.862 (0.361-58.271)	0.365	71472865.597 (0.000-NA)	0.995
M stage (M1 vs. M0)	1.000 (0.119-8.433)	1.000	65432904.513 (0.000-NA)	0.994
Pathologic stage (stage III & stage IV vs. stage I & stage II)	1.862 (1.147-3.056)	0.013	1.805 (1.112-2.962)	0.018
Gender (male vs. female)	0.417 (0.265-0.650)	<0.001	0.376 (0.238-0.587)	<0.001
Age (>60 vs. ≤60)	1.396 (0.929-2.102)	0.109	0.657 (0.436-0.987)	0.044
BMI (>25 vs. ≤25)	1.030 (0.671-1.580)	0.894	0.543 (0.352-0.836)	0.006
AFP (ng/ml) (>400 vs. ≤400)	1.589 (0.910-2.805)	0.106	3.922 (2.155-7.432)	<0.001
Albumin (g/dl) (≥3.5 vs. <3.5)	0.814 (0.473-1.394)	0.454	1.775 (1.027-3.124)	0.042
Vascular invasion (yes vs. no)	1.002 (0.631-1.592)	0.993	1.427 (0.898-2.276)	0.133
Child-Pugh grade (B vs. A)	0.876 (0.345-2.154)	0.775	0.553 (0.203-1.383)	0.219

**(b):** 

Characteristics	VEGFC		VEGFD	
	Odds ratio (OR)	*P* value	Odds ratio (OR)	*P* value
T stage (T2 & T3 & T4 vs. T1)	0.870 (0.578-1.307)	0.501	1.493 (0.992-2.251)	0.055
N stage (N1 vs. N0)	2.907 (0.367-59.196)	0.358	1.032 (0.122-8.708)	0.975
M stage (M1 vs. M0)	3.185 (0.402-64.826)	0.318	1.078 (0.128-9.087)	0.941
Pathologic stage (stage III & stage IV vs. stage I & stage II)	0.915 (0.565-1.478)	0.716	1.645 (1.015-2.692)	0.045
Gender (male vs. female)	0.885 (0.573-1.365)	0.581	1.130 (0.733-1.745)	0.581
Age (>60 vs. ≤60)	0.781 (0.519-1.173)	0.234	1.776 (1.180-2.684)	0.006
BMI (>25 vs. ≤25)	1.167 (0.761-1.792)	0.480	1.520 (0.990-2.341)	0.056
AFP (ng/ml) (>400 vs. ≤400)	0.564 (0.317-0.989)	0.048	0.887 (0.507-1.545)	0.671
Albumin (g/dl) (≥3.5 vs. <3.5)	1.430 (0.834-2.471)	0.195	0.872 (0.507-1.495)	0.620
Vascular invasion (yes vs. no)	0.757 (0.475-1.202)	0.239	1.344 (0.846-2.144)	0.211
Child-Pugh grade (B vs. A)	0.310 (0.099-0.822)	0.027	1.090 (0.442-2.717)	0.851

**Table 3:** Characterization of VEGF gene expression in AD.

Characteristic	Control	AD	*P* value
Number	530	204	
Sex, *n* (%)			0.29
Female	295 (40.2%)	104 (14.2%)	
Male	235 (32%)	100 (13.6%)	
Age	73 (68, 77)	72 (67.75, 79)	0.893
Connectivity *z* score, median (IQR)	0.28 (-0.5, 0.67)	0.37 (-0.18, 0.65)	0.166
Batch, median (IQR)	32 (23, 37)	33 (30, 37)	0.097
VEGFA, median (IQR)	7.49 (7.38, 7.52)	7.38 (7.32, 7.48)	<0.001
VEGFB, median (IQR)	7.45 (7.3, 7.49)	7.29 (7.27, 7.34)	<0.001
VEGFC, median (IQR)	7.47 (7.33, 7.51)	7.33 (7.3, 7.37)	<0.001

## Data Availability

Transcriptomic data and clinical data for patients with HCC were downloaded from the TCGA database (https://portal.gdc.cancer.gov). The human cognitive impairment-related dataset GSE140831 was obtained from the GEO database in NCBI.

## Abbreviations

VEGF: Vascular endothelial growth factor
AD: Alzheimer's disease
ROC: Receiver operating characteristic curve
AUC: Area under the curve.
